# Analyzing the Role of Corporate Social Responsibility for Sustainable Environmental Performance: Mediating Roles of Environmental Strategy and Environmental Outcomes

**DOI:** 10.3389/fpsyg.2022.906610

**Published:** 2022-06-23

**Authors:** Xiaodong Wang, Weijun Bian

**Affiliations:** ^1^School of Humanities and Social Sciences, Xi’an Jiaotong University, Xi’an, China; ^2^School of Literature and Business, Xi’an Siyuan University, Xi’an, China

**Keywords:** corporate social responsibility, environmental outcomes, environmental strategy, SMEs, China

## Abstract

This study examines the relationship between corporate social responsibility (CSR) and environmental performance, utilizing data from 415 small and medium-sized enterprises (SMEs) in China as a case study. We found that CSR has a direct and significant impact on environmental performance (EP) and is positively correlated to environmental strategy (ES) and environmental outcomes (EO), both of which improve environmental performance, i.e., they serve as a significant mediating factor between CSR and environmental performance. Our study will help general managers and policy maker of SMEs, provides a beneficial model for managing CSR, ES, and EO to achieve sustainable environmental performance. Specifically, it can assist general managers of SMEs in strengthening their internal resources such as CSR, ES, and EO in order to improve long-term environmental performance.

## Introduction

Authors have recently become increasingly interested in the connection between environmental performance and corporate social responsibility (CSR). It’s hard to say for sure, though, because some studies found a positive correlation between CSR and environmental performance, while others found either a negative correlation or no correlation at all. Recent research of CRS in industrial firms has just begun. Many of these studies focus on how CRS affects environmental performance directly (Kraus et al., 2020).

Chuang and Huang (2018) examined the direct relationship between corporate social responsibility and environmental performance in order to discover whether it has a beneficial or negative impact on the environment. While some studies (i.e., Delmas et al., 2013) have discovered a link between the two, others have suggested that the relationship could be influenced by other factors not considered in the research. According to Karassin and Bar-Haim (2019), there is no direct relationship between corporate social responsibility and environmental performance. The firm’s intangible resources, on the other hand, were utilized to mediate the relationship. There has been an upsurge in research and practice linking corporate social responsibility and environmental strategy as a result of the renewed interest in employee-focused corporate social responsibility and environmental strategy (Channa et al., 2021; Jamil et al., 2021a). Corporations’ social responsibility (CSR) and environmental performance are interwoven, with environmental strategy having an impact on the formulation and implementation of CSR programs.

Also relevant are the concepts of corporate social responsibility (CSR) and environmental performance, which can be seen as complementary when it comes to understanding assumptions about not only the role of corporations, but also the relationship between organizations and the environment (Anser et al., 2020; Awan et al., 2022). The fact that calls are being made for more research into the relationship between corporate social responsibility, environmental strategy, and environmental outcomes should not come as a surprise, since, while research has certainly begun to pay greater attention to this connection, a more comprehensive examination of the relationship between these two constructs has yet to be undertaken, particularly with regard to the potential link between environment and corporate social responsibility (Nassani et al., 2022). We believe that such an endeavor is highly important and vital because there are various significant interactions between the environment and corporate social responsibility (CSR) that have not been sufficiently or systematically addressed.

As a result, the relationship between corporate social responsibility and environmental performance is arguably more complicated than what the findings of many previous studies suggest (García Martín and Herrero, 2020; Peng et al., 2021); as a result, we decided to use this study as a means of expanding the scope of previous research works on the link between corporate social responsibility and environmental performance within Chinese manufacturing firms. New research questions will be asked with this aim in mind: Do CSR has impact on environmental performance? and ‘Do environmental strategy and environmental outcomes (EOs) act as mediators in the relationship between CSR and environmental?’

Our findings make a number of important contributions to the fields of corporate social responsibility and the environment. For the former, this study not only makes it easier to resolve some of the ambiguity surrounding the relationship between CSR and environmental performance, but it also contributes to the expansion of CSR knowledge through the development of an explanation for the possible association between CSR and environmental performance through the inclusion of environmental sustainability and environmental performance indicators (ES and EOs) as mediating variables. In addition, corporate social responsibility (CSR) occurs as an antecedent aspect in strategy. An existing gap in the literature about the effects of environmental strategy on environmental performance was filled by concluding that environmental outcomes had a positive impact on environmental performance, which was previously undiscovered.

After the introduction section literature review in discussed with relevant theory after that research methodology and results of the study are presented. Next section is discussion of results with implications of the study and at the end limitations and future research directions are discussed.

## Literature Review and Hypotheses Development

### Natural Resource-Based View Theory

Organizational resources and competencies are critical to long-term competitive advantage, according to RBV theory (Hart, 1995). RBV theory’s extended variation, the natural RBV theory, proposes that firms could benefit from a long-term competitive advantage if they respond quickly to environmental issues. RBV theory is lacking in a number of ways, according to (Hart, 1995). The relationship between the organization’s natural surroundings and the organization itself is not taken into account, among other factors. Although this exclusion may have been warranted in the past, nature’s role in the marketplace has become increasingly obvious. Hart and Dowell (2011) found that reducing pollution through the use of natural resources and capabilities leads to an improvement in profitability. Additional factors that contribute to increased long-term performance and sustainability include environmental resources, pollution prevention strategies, and organizational competences. In order to evaluate a company’s social responsibility, researchers might use natural RBV theory to focus on environmental, social, and economic aspects of CSR (Úbeda-García et al., 2021). Stakeholder theory was used in past research on CSR and economic performance and ability motivation-opportunity theory was used in previous studies on environmental strategy and environmental management performance (Partalidou et al., 2020). Natural RBV theory was used by the researchers to lessen the emphasis on measuring environmental performance through CSR, environmental outcomes, and environmental strategy. For this study, researchers looked at the role of environmental outcomes as well as the role of CSR in enhancing environmental performance.

### Corporate Social Responsibility, Environmental Strategy and Environmental Performance

For the past few years, professionals have focused their attention on corporate social responsibility (CSR) since consumers want environmentally friendly products and services. Someone who is concerned about environmental issues in a number of businesses, as well as the introduction of environmentally-friendly products and procedures into the market is an “eco-entrepreneur.” Competition, consumers, employees, and the government have all put pressure on a number of companies to speak out on social and environmental issues. Corporations throughout the world have begun to practice CSR in recent years (Bhalla and Overton, 2019; Gul et al., 2021a). Despite the fact that numerous studies have been conducted on CSR, there is no commonly acknowledged definition of the term (Aragón-Correa et al., 2008; Cha et al., 2019). A study of this nature proved difficult for the researchers, as a result. If a company is to be successful, it must meet the expectations of the broader public. A company’s life expectancy is shorter when it is internally focused, whereas companies that put the needs of their customers first are more likely to succeed in today’s market (Orazalin and Baydauletov, 2020). An organization’s commitment to pursuing strategies, making decisions, and doing actions that benefit society at large is known as corporate social responsibility (CSR). Corporate social responsibility (CSR) encompasses economic, social, and environmental considerations. Research examining the link between CSR and organizational performance is rare, but what little research there is shows that CSR boosts performance. According to Grubor et al. (2020) Corporate social responsibility (CSR) is becoming an increasingly significant part of business. Researchers have studied the link between corporate social responsibility and economic performance in micro, small, and medium-sized businesses and found that CSR significantly enhances economic performance (Sila and Cek, 2017; Marakova et al., 2021). As a result, academics focused primarily on assessing the environmental performance of these enterprises without paying much attention to corporate social responsibility (CSR). Here, our investigation aims to fill the gap.” Therefore, following hypothesis proposed:

**H1:** CSR relates to SEP.

**H2:** CSR relates to ES.

### Environmental Strategy, Environmental Performance

RBV theory doesn’t take environmental strategy into account when analyzing the success of businesses. Natural RBV theory, on the other hand, placed greater focus on environmental sustainability as a means of gauging long-term viability. Scholars and practitioners are mostly focused on environmental strategy (Rodrigue et al., 2013; Jamil et al., 2021b). It has been found that companies that have environmental plans are more likely to realize environmental advantages than those who do not (Xie et al., 2020). Organizational resources or strategic positioning should be used to evaluate an organization’s success, according to experts (Chen et al., 2015). This is a point of contention. Business strategy has recently been discovered to be an important predictor in environmental protection and economic operations. Furthermore, research shows that taking a pro-active approach to environmental issues boosts a company’s long-term financial and economic performance (Samad, 2018). Some of the environmental projects also looked into how organizations performed (Latan et al., 2018; Awan et al., 2021). The performance of management is unaffected by environmental measures. There is a lack of clear evidence to support the link between business strategy and corporate performance.

**H3:** ES relates to SEP.

### Corporate Social Responsibility and Environmental Outcomes

What constitutes a company’s responsibility toward the environment and its operating parameters is defined in terms of environmental outcomes. CSR practices and environmental consequences have already been studied in earlier research, with a variety of studies looking into subjects such as the relationship between CSR and green supply chain management, individual green behavior, and employee environmental engagement. The literature on corporate social responsibility has been examined in addition to quantitative research (Aleksić et al., 2020; Gul et al., 2021b).

Consequently, corporate social responsibility (CSR) may be a significant issue to consider for improving environmental effects. This means that it is easier to describe the environmental repercussions of particular corporate social responsibility activities (Huang, 2010). Evaluation of green performance by employees in the same vein helps to align behavior and accountability and place a higher emphasis on environmental objectives all of which contribute to better environmental results for business (Ko and Liu, 2017; Rozsa et al., 2021). Environmentally friendly activities can be put to use by employees who have a strong emphasis on employee involvement, as well as innovative solutions to waste reduction and resource utilization efficiency improvement in the workplace, all of which contribute to the improvement of the company’s environmental outcomes. When CSR is correctly applied, it has the ability to improve environmental performance (Shaukat et al., 2016; Jamil et al., 2022).

**H4:** CSR relates to EO.

### Environmental Outcomes and Environmental Performance

The hypotheses made by Porter, Van der Linde, and Hart (1995) have led to more support for the idea that environmental management can be used to gain a competitive advantage. At the same time, some people aren’t so sure (Peng et al., 2021). For example, a lot of research has shown that improving the environment would lead to better performance, which shows that there is a link between these two variables. Companies that care about the environment will be more credible and successful at meeting the needs of their stakeholders, which will lead to a better corporate image, less tax, and less environmental costs for the company (Latan et al., 2018).

To this point, there hasn’t been a clear answer to the question of whether or not better environmental results will lead to better financial results (Shaukat et al., 2016). In order to get better environmental results, you’ll have to spend more money on things like risk management or more money for things like capital and operations and energy (Sila and Cek, 2017). This means that your overall performance will be lower. Environmental outcomes, on the other hand, can lead to more market access and better product differentiation, which can lead to better performance.

**H5:** EO relates to SEP.

### Mediating Role of Environmental Strategy and Environmental Outcomes

Environmental strategy and environmental outcomes are influenced by CSR as a result of CSR, and thus leads to improved environmental performance, as was previously discussed in the context of corporate social responsibility (Cho et al., 2019). Studies have shown that corporate responsibility (CSR) significantly improves organizational performance. In spite of this, Solovida and Latan (2017) found that there is a mixed association between corporate social responsibility and economic performance (Partalidou et al., 2020). Thus, the relationship between corporate social responsibility and business performance is ambiguous and requires more examination by incorporating a mediating component into the equation. In Hart (1995), the natural RBV theory, the link between environmental resources and competitive advantage is attributed to environmental strategy and environmental outcomes (Ryszko, 2016). Environmental strategy and results are used to mediate the relationship between environmental performance and corporate social responsibility.

**H6:** ES mediates the relationship of CSR and SEP.

**H7:** EO mediates the relationship of CSR and SEP.

## Conceptual Framework



### Research Methodology

In this study, we collected information from small and medium-sized firms (SMEs) in five of China’s largest industrial cities. A convenient sampling strategy was used in this study (Kothari, 2004). Employees were asked to complete a questionnaire in English, and a translation into Chinese was also provided on the questionnaire for better understanding by those who responded. The total number of participants in this study was 415 middle and upper-level executives from various businesses. There was a total of 625 questionnaires circulated by email, with 445 responses receiving the most attention. According to the final analysis, a total of 415 appropriate responses were received, representing a response rate of 71.2 percent. Data from a survey is cleaned to remove responses from people who don’t meet our target requirements or who didn’t respond carefully to the questionnaire survey, like people who only answer part of the survey, people who give ambiguous answers or choose the same answer option over and over again, and people who give incomprehensible suggestions for open-ended questions. Valid questionnaires are chosen after the survey data cleaning process, which involves removing responses from respondents who either don’t meet our target requirements or don’t meet our target requirements. We used Armstrong and Overton (1977) method for anti-reaction bias. An independent sample and chi-square T-tests were used to compare and contrast the first 45 and last 45 people who took the survey based on their age and gender. The data showed that there were no big differences between the two answer groups (*p* > 0.05).

### Variable Selection and Process

The study used items established from prior research to confirm the reliability and validity of the measures. All items are evaluated through five-point Likert-type scales where “1” (strongly disagree), “3” (neutral), and “5” (strongly agree).

*Dependent Variable:* To get response about sustainable environmental performance we used five items adopted from the prior study of (Laosirihongthong et al., 2013).

*Independent variable:* To analyze corporate social responsibility with its three dimensions we used eleven items adopted from prior study of Alvarado-Herrera et al. (2017) and detail of items are following:

1. CSR toward society is determined by four-items and the sample item is, “Our organization emphasizes the importance of its social responsibilities before society.”
2. CSR toward customers is determined by three-items and the sample item is, “Customer satisfaction is a priority for our organization.”
3. CSR toward employees is determined by four-items and the sample item is, “Our organization implements flexible policies to provide a good work & life balance for its employees.”

*Mediating variables:* Environmental strategy and environmental outcomes are used as mediating variables. Environmental strategy was measured with four items adopted from Banerjee (2002), and sample item is, “Our firm has integrated environmental issues into our strategic planning process,” while environmental outcomes is measured with five items adopted from Zailani et al. (2014) and the sample item is, “Reduction of total direct and indirect toxic emissions.”

### Sample Description

The demographic profile of 415 respondents, such as ownership form of the organization, age of the organization and size of the organization, are shown in Table 1.

**TABLE 1:** Characteristics of the respondents.

*Characteristics*	*Range*	*Frequency*	*Percentage*
Age of Organization	Less than 10 years	60	14.45%
	10-20 years	95	22.90%
	20-30 years	135	32.50%
	Above 30 years	125	30.15%
	**Total**	**415**	**100.00%**
Ownership of Organization	Government Owned	160	38.50%
	Private Owned	265	61.50%
	**Total**	**415**	**100.00%**
Size of Organization	Less than 100 employees	103	28.80%
	100-200 employees	97	23.37%
	200-300 employees	111	26.74%
	More than 300 employees	104	21.09%
	**Total**	**415**	**100.00%**

## Results

This study used smart PLS to evaluate the model. This study wants to use confirmatory and exploratory research so the PLS-SEM analysis was selected. Sarstedt et al. (2014) argue that Behind the Partial least square modeling, there are two approaches known as structural modeling and covariance biased. The hypothesis testing was done through PLS-SEM and the hypothesis expansions was usually tested through SEM (Hair et al., 2016). The PLS is best suited for multi constructs model and multiple order constructs models. The small sample size is used for analysis is also advantageous in Smart PLS-SEM. Smart PLS-SEM provides it straightforward to compute all parameter computations (Hair et al., 2016). The current study was done using Smart PLS 3.9.

The degree to which the study variables deviate from their latent variable is called unidimensional. In order to verify construct reliability and validity, an investigation of the study constructs’ unidimensional is a criterion that must be achieved (Chou et al., 2007). According to Byrne (2001), the factor loading of items within each construct was used to determine unidimensional. There is strong evidence that all of the constructs indicated in the measurement model are unidimensional (Usman Shehzad et al., 2022).

### Model Measurement

The study is quantitative in nature and data was collected through survey questionnaire. The study analyzed the corporate social responsibility on sustainable environmental performance through the mediating role of environmental safety and outcome. Firstly, we examine the construct reliability and validity of the external model through Smart PLS algorithm (Table 2 and Figure 1). Factor loading and Cronbach Alpha was used to assess the model reliability, The analysis show that 24 indicators out of 28 have factor loading greater than 0.6 which meet the model reliability (Hair et al., 2016). Cronbach’s alpha, Average variance extracted and composite reliability may be used to determine the degree of consistency between several measurements of a variable (Hair et al., 2010). The value of Cronbach Alpha for all variables should be greater than threshold level which is 0.7 (Hair et al., 2014). The factor loading of 24 indicators is greater than 0.7, Cronbach’s alpha (α) for all constructs meet the acceptable threshold level which is 0.7. On the other hand the composite reliability for all constructs exceed the threshold level 0.70 which meet the minimum acceptable criteria (Chin, 1998; Bagozzi et al., 1991). Composite reliability values ranged from 0.81-0.903 and were all above the recommended value which is 0.6 (Bagozzi and Yi, 1988) or greater than 0.70 as suggested byy Holmes-Smith (2001). In light of these findings, it can be concluded that all of the research hypotheses examined in this study are valid and trustworthy. The factor loading, Cronbach’s alpha (α), a composite reliability confirms the indicator reliability (Chin, 1998; Henseler et al., 2009).

**TABLE 2:** Inner model evaluation.

Variables	Constructs	Factor loading	Cronbach’s Alpha	Composite reliability	Average variance extracted (AVE)
**Corporate Social Responsibility**					
CSR Customer	CSRC2	0.883	0.710	0.873	0.775
	CSRC3	0.878	0.745	0.897	0.835
*CSR for*	CSRE1	0.780	0.736	0.851	0.655
*Employees*	CSRE2	0.798			
	CSRE3	0.848			
*CSR for society*	CSRS1	0.718	0.803	0.872	0.633
	CSRS2	0.692			
	CSRS3	0.883			
	CSRS4	0.871			
*Environmental*	EO1	0.712	0.809	0.860	0.552
*sustainability*	EO2	0.753			
	EO3	0.762			
	EO4	0.734			
	EO5	0.752			
*Environmental*	EP1	0.664	0.870	0.903	0.609
*performance*	EP2	0.774			
	EP3	0.847			
	EP4	0.778			
	EP5	0.773			
	EP6	0.834			
*Environmental*	ES1	0.816	0.825	0.884	0.656
*strategy*	ES2	0.772			
	ES3	0.827			
	ES4	0.822			

**FIGURE 1:** Bootstrapping.

The convergent validity of variables is evaluated by using the “composite reliability” (CR) and “Average variance extracted” (AVE), and construct reliability for all variable (Hair et al., 2016). The researchers say that CR and AVE must should be higher than the minimum acceptable value which is 0.7 and 0.5 consecutively. By utilizing composite reliability and average variance extracted (Fornell and Larcker, 1981a). The Table 3 indicate that all variables have loading higher than 0.70 and CR is greater or equal to 0.70, The AVE score should be greater than 0.50 which illustrate the convergent validity is acceptable and internal consistency of items (Hair et al., 1998: Chinand Newsted, 1999).

**TABLE 3:** Discriminant validity: Fornell-Larcker criterion.

	CSRC	CSRE	CSRS	CSR	ES	EO	SEP
CSRC	0.881						
CSRE	0.692	0.809					
CSRS	0.755	0.736	0.796				
CSR	0.870	0.790	0.736	0.733			
ES	0.639	0.803	0.604	0.639	0.810		
EO	0.508	0.561	0.708	0.670	0.721	0.743	
SEP	0.627	0.789	0.788	0.728	0.773	0.694	0.780

*Note: CSR customers (CSRC); CSR employees (CSRE); CSR society (CSRS); Corporate social responsibility (CSR); Environmental strategy (ES); Environmental Outcome (EO); Sustainable Environmental Performance (SEP).*

### Discriminant Validity

Several tests were used to examine discriminant validity. As a first step, it may be explored in the measurement model by looking at the latent constructs’ shared AVE. To determine whether of the model is evaluated through the correlation among constructs. If there are any extremely high correlations among constructs, the model is likely to have discriminant validity issues. Construct validity occurs when the square correlation for each construct surpasses the AVE for each of the other components (Fornell and Larcker, 1981b). AVE values for each construction were more than or equal to 0.50, as shown in Table 4, indicating that the values ranging from 0.54 to 0.71 were responsible for more than half of the variation in their respective measurement items, as recommended. Fornell–Larcker criteria and heterotrait–monotrait (HTMT) ratio are two strategies used to assess the discriminant validity of the model (Hair et al., 2016). the Fornell and Larcker (1981b) argue that it’s important to keep in mind that upper right side values of the diagonal which is the square root of AVE should be larger than the correlation with other constructs (Fornell and Larcker, 1981b; Hair et al., 2016). However, values between 0.90 and 0.95 are acceptable for HTMT ratios but must be less than 0.85 (Hair et al., 2016). There are no HTMT ratios greater than 0.90 in Table 3, confirming the discriminant validity of the model.

**TABLE 4:** Hypothesis testing.

	Hypothesis	Original sample (O)	Sample mean (M)	Standard deviation (STDEV)	T statistics (| O/STDEV|)	*P* values
H1	CSR - > SEP	0.301	0.306	0.071	4.219	0.000
H2	CSR - > ES	0.839	0.836	0.028	29.984	0.000
H3	ES - > SEP	0.554	0.543	0.074	7.474	0.000
H4	CSR - > EO	0.670	0.671	0.041	16.349	0.000
H5	EO - > SEP	0.093	0.101	0.046	2.036	0.042

*Corporate social responsibility has positive and significant impact on environmental Outcome (β = 0.670, t value = 16.349, p-value = 0.000). Environmental outcome has significant impact on sustainable environmental performance (β = 0.093, t-value = 2.036, p = 0.042). The findings indicate the Hypothesis H1, H2, H3, H4 and H5 are accepted.*

The Variance Inflation factor (VIF), values were computed in this study to check for Conceptual model collinearity concerns. VIF values below 5 indicate that no collinearity issues exist in the data, according to experts (Hair et al., 2014). It was found that the objects’ inner VIFs ranged from 1.321 up to 1.876. The results of this investigation show that there is no evidence of data collinearity, and that the conclusions remain constant throughout time. All of the model’s latent variables have Q2 values suggest that model is highly predictive (Hair et al., 2014; Mohsin et al., 2021).

R2 greater than 0.5 indicates a suitable model. All exogenous constructs have R Squared values larger than 0.5 in Figure 2, indicating that the model’s predictive accuracy is quite high (Hair et al., 2016).

**FIGURE 2:** Composite reliability.

When assessing the model’s “explanatory power,” the R2 value for each predicted variable was computed. it indicated that the degree to which the IV explains the DV. Predictive accuracy is measured by the R2 value, which ranges from 0 to 1. R2 value described as “weak,” “moderate,” and “strong,” with R2 describe as week with value 0.25 and R2 value is moderate with 0.50. and R2 value is 0.75 considered as substantial. All exogenous constructs in Table 5 have R Square values higher than 0.5, except environmental strategy which indicates that the model has moderate predictive accuracy (Hair et al., 2016; Li et al., 2021).

**TABLE 5:** Predictive accuracy.

	R square	R square adjusted
Environmental strategy	0.704	0.703
environmental outcome	0.449	0.447
sustainable environmental performance	0.798	0.796

### Model Assessment

This study examines the hypothesis by using bootstrapping at 5000 with sample replacement (Hair et al., 2016). The results show that corporate social sustainability has positive and significant impact on sustainable environmental performance (β = 0.301, *t* value = 4.219, *p*-value = 0.000). corporate social sustainability has positive and significant impact on environmental strategy (β = 0.839, *t* value = 29.984, *p*-value = 0.000). Environmental strategy has positive and significant impact on sustainable environmental performance (β = 0.554, *t* value = 7.474, *p*-value = 0.000).

### Mediation Analysis

Environmental strategy mediates the relationship between CSR and sustainable environmental performance. the value for VAF greater than 80 percent suggest full mediation, whereas VAF greater than 20% and higher than 80% show partial mediation, and VAF less than 20 percent indicates no mediation. The findings indicate that environmental strategy partially mediate the relationship between corporate social responsibility and sustainable environmental performance. There was an indirect impact (beta = 0.465, *t*-value = 7.939, *p*-value = 0.000) with VAF 76 percent, which indicates partial mediation. The findings indicate that environmental outcome partially mediate the relationship between corporate social responsibility and sustainable environmental performance (beta = 0.062, *t*-value = 2.129, *p*-value = 0.000) with VAF 62 percent, which indicates partial mediation VAF is used to indicate the amount of the indirect impact relative to overall effects, and it is calculated as a percentage of total effects. Partially mediating the impact of both the direct and indirect effects (Zhao et al., 2010; Nitzl et al., 2016) (see Table 6 for all mediating relationships).

**TABLE 6:** Mediation analysis.

Hypothesis	Direct effect	Indirect effect	Total Effect	VAF	Explanation	Result
CSR - > ES - > SEP	0.301 (4.219)	0.465 (7.939)	0.828 (24.921)	68%	Partial Mediation	H6, Supported
CSR - > EO - > SEP	0.301 (4.219)	0.062 (2.129)	0.432 (11.34)	72%	Partial mediation	H7 supported

## Discussion and Conclusion

This article’s CSR framework considers environmental strategies for Chinese manufacturing SMEs. According to the findings, CSR has an impact on environmental performance. There is a strong correlation between corporate social responsibility and business performance, according to Cho et al. (2019). On the other hand, Anser et al. (2020) contradicted this finding that a company’s performance is evaluated by its CSR initiatives. Environmental strategies have a substantial impact on the long-term performance of an organization, according to the natural RBV theory (Hart, 1995). According to Martinez-Conesa et al. (2017) CSR has a substantial impact on a company’s financial performance and managers and owners can’t ignore it. CSR has a significant impact on environmental strategy. According to Martinez-Conesa et al. (2017) when confronted with environmental, economic, and social constraints, a company’s business model and strategy may be better aligned. This research to see how corporate social responsibility affects environmental performance. During the investigation, a gap was discovered. CSR is having a huge impact on the environment and how it affects the ecosystem while this is going on. Environmental CSR and environmental strategy have a glaring omission from much of the existing literature (Karassin and Bar-Haim, 2019). We see a link between corporate social responsibility (CSR) and environmental results that most academics do not, and we intend to change that.

The environmental strategy has a significant impact on the effectiveness of the environmental performance. Channa et al. (2021), for example, discovered that environmental strategy can have a significant impact on environmental performance and Sari and Tjen (2017) also discovered that, contrary to widespread perception, environmental strategies have little impact on how managers are rated. As indicated by the statistics, environmental approaches have a major impact on long-term performance, which is in accordance with the natural RBV theory (Hart, 1995; Hart and Dowell, 2011). When determining a company’s success, RBV theory does not take into consideration the business plan of the company. When it comes to enhancing environmental performance, Hart (1995) was the first to recognize the role of corporate strategy, specifically environmental strategy, in the process. Another aspect that determines environmental performance is the environmental performance of a company’s operations. Úbeda-García et al. (2021) argue that businesses can gain a competitive advantage by enhancing their environmental performance. The RBV theory is correct in the sense that long-term performance can be improved by introducing new ideas (Hart, 1995).

The environmental strategy and environmental outcomes serve as a mediating between corporate social responsibility and environmental performance. We believe that corporate social responsibility has a direct impact on environmental performance, as well as an indirect impact on environmental performance through environmental strategy and environmental outcomes (Wang and Sarkis, 2017). The natural RBV hypothesis proposes that corporate social responsibility (CSR) is linked to environmental strategy and outcome in the same way that environmental performance is linked to CSR. At the end, we discovered that corporate social responsibility has a direct impact on environmental performance. The majority of the time, corporate social responsibility has a significant impact on environmental strategy and outcomes (Xie et al., 2020). Lower emissions, lower energy consumption, lower raw material consumption, and lower usage of hazardous materials are all benefits of the environmental plan and its implementation, according to the results. Finally, environmental performance and corporate social responsibility are intertwined through environmental strategy and results.

## Theoretical Implications

It is necessary to unearth research findings that can shed light on a significant organizational issue in order to make a theoretical Contribution To The Field. Another essential component of our research is that it offers a fresh viewpoint on corporate social responsibility (CSR), environmental strategy, ecological outcomes and ecological performance. This is one of the most important aspects of our research. There is a link between CSR and EP, as well as between the function of environmental strategy and its consequences and their application in the mediation process (Rodrigue et al., 2013). As a result, our research is a ground-breaking study in that it brings together CSR, ES, EO, and environmental performance into a single research model that is unprecedented. We are pleased with the contribution we have made to these fields (Naseem et al., 2021). All of these theories have been used in the past to analyze (CSR), environmental strategy, environmental outcomes, and environmental performance. When evaluating the influence of CSR on economic performance, for example, stakeholder theory can be utilized to make inferences. It was based on the ability motivation opportunity paradigm that a second line of research was conducted, which focused on EP. A contingency theory approach was utilized to examine the relationship between environmental strategy and environmental management performance.

## Practical Implications

Our findings should be taken into consideration by management consultants and lawmakers. We’ve developed a research technique to assist large industrial organizations in better understanding the relationship between corporate social responsibility, environmental strategy, and green innovation. This technique is intended to steer them in the proper way. Higher management of the organization is concerned about EP in today’s world; nevertheless, they may benefit from the study outcomes related to EP which will helpfully make policies to minimize wastage and air pollution. Although the relationship between CSR and environmental performance has evolved as a result of environmental strategy and results, there is no direct link between the two. Since various studies have demonstrated that CSR has a significant impact on organizational performance, general managers of large industrial organizations should not disregard CSR while analyzing environmental performance in their organizations (Chen et al., 2015). CSR, ES, and EO must be given top priority by general management and policymakers in order to assess environmental performance.

## Limitations and Future Research Directions

Even if it contains some of the same limitations as prior studies, these flaws can be addressed by other researchers in the future. Starting with a cross-sectional perspective, experts aren’t sure whether corporate social responsibility, environmental strategy, and green innovation in large industrial organizations will continue to work in the same way over time. The same research framework will be used by future researchers to see whether or not the results remain consistent over a longer period of time. Future studies can look at data from small and medium-sized firms in China to observe how the outcomes vary over time, much as our study looked at data from small and medium-sized enterprises in China. The function of green competence and green transformational leadership as a relationship between corporate social responsibility and environmental performance can also be investigated by future scholars. Finally, the current research was carried out in China, which has its own culture and traditions. It will be possible for future researchers to replicate the study in other nations to discover whether there are any changes. In addition, concepts from the circular economy can be applied to the evaluation of social, environmental, and economic performance outcomes.

## Data Availability Statement

The raw data supporting the conclusions of this article will be made available by the authors, without undue reservation.

## Author Contributions

Both authors listed have made a substantial, direct, and intellectual contribution to the work, and approved it for publication.

## Conflict of Interest

The authors declare that the research was conducted in the absence of any commercial or financial relationships that could be construed as a potential conflict of interest.

## Publisher’s Note

All claims expressed in this article are solely those of the authors and do not necessarily represent those of their affiliated organizations, or those of the publisher, the editors and the reviewers. Any product that may be evaluated in this article, or claim that may be made by its manufacturer, is not guaranteed or endorsed by the publisher.
